The article "Lipolytic Potential of Aspergillus japonicus LAB01: Production, Partial Purification, and Characterisation of an Extracellular Lipase" was published in 2014. Journal: Biomed Res Int.

# Lipolytic Potential of *Aspergillus japonicus* LAB01: Production, Partial Purification, and Characterisation of an Extracellular Lipase

**DOI:** 10.1155/2014/108913

**Published:** 2014-10-29

**Authors:** Lívia Tereza Andrade Souza, Jamil S. Oliveira, Vera L. dos Santos, Wiliam C. B. Regis, Marcelo M. Santoro, Rodrigo R. Resende

**Affiliations:** ^1^Cell Signaling, Nanobiotechnology and Enzymology Laboratory, Federal University of Minas Gerais, 31270-901 Belo Horizonte, MG, Brazil; ^2^Laboratory of Applied Microbiology, Federal University of Minas Gerais 31270-901, Belo Horizonte, MG, Brazil

## Abstract

Lipolytic potential of* Aspergillus japonicus *LAB01 was investigated by describing the catalytic properties and stability of a secreted extracellular lipase. Enzyme production was considered high under room temperature after 4 days using sunflower oil and a combination of casein with sodium nitrate. Lipase was partially purified by 3.9-fold, resulting in a 44.2% yield using ammonium sulphate precipitation (60%) quantified with Superose 12 HR gel filtration chromatography. The activity of the enzyme was maximised at pH 8.5, and the enzyme demonstrated stability under alkaline conditions. The optimum temperature was found to be 45°C, and the enzyme was stable for up to 100 minutes, with more than 80% of initial activity remaining after incubation at this temperature. Partially purified enzyme showed reasonable stability with triton X-100 and was activated in the presence of organic solvents (toluene, hexane, and methanol). Among the tested ions, only Cu^2+^, Ni^2+^, and Al^3+^ showed inhibitory effects. Substrate specificity of the lipase was higher for C14 among various p-nitrophenyl esters assayed. The K_M_ and *V*_max_ values of the purified enzyme for p-nitrophenyl palmitate were 0.13 mM and 12.58 umol/(L*·*min), respectively. These features render a novel biocatalyst for industrial applications.

## 1. Introduction

*Aspergillus japonicus* is amenable for biotechnological analysis due to its phytase [1], cellulose [2], pectinase [3], xylanase [4, 5], and beta-fructofuranosidase [6] production capacity. Furthermore, the production of fibrolytic enzymes is well described; however, their lipolytic potential remains unknown. Lipases (triacylglycerol hydrolases, EC.3.1.1.3) are a class of serine hydrolases that belong to the *α*/*β* hydrolase super family. Depending on the water activity and the tolerance of organic solvents, lipases can act as modifying triacylglycerides by catalysing hydrolysis and different synthetic reactions, such as esterification, interesterification, and transesterification, with different specificities, efficiencies, and environmental compatibilities [7]. Interestingly, direct correlations between the enzyme activities in aqueous or organic media are lacking. Thus, some lipases have significant potential for application in oil and fat hydrolysis, but almost none have been applied in industrial processes, such as biodiesel production [8]. Reaction versatility is an important feature of this enzyme and is a subject to be investigated in the search for new lipases.

The article "Lipolytic Potential of Aspergillus japonicus LAB01: Production, Partial Purification, and Characterisation of an Extracellular Lipase" was published in 2014. Journal: Biomed Res Int.

Lipases are regarded as the most important enzymes for biocatalysis in organic media and have been industrially used as lipid stain digesters in detergent formulation, the preparation of various products, and aromas in the food industry, structured lipids synthesis, leather processing, enantioresolution esters for chemical and drug intermediates, biodiesel production, and the treatment of waste products rich in oil [9].

Most industrial microbial lipases are derived from fungi, especially the* Aspergillus *genus [10]. Over the years, efforts have been directed to describe lipases from a variety of species, including* A. nomius* [11],* A. niger* [12],* A. carneus* [13],* A. repens* [14],* A. terreus* [15, 16],* A. oryzae* [17], and* A. wentii* [18]. In general, lipases obtained from* Aspergillus *are promising for their catalytic properties, such as thermal stability, specificity, stereospecificity, tolerance of organic solvents, and bulk production [10].

Lipases have emerged as leading biocatalysts, with less than 5% of participation in the global market; the market is expected to grow over the coming years, mainly due to the application of enzymes in the biofuel industry (biodiesel). Due to the increase in the biotechnological importance and potential of enzymes to contribute to the multibillion dollar unexploited bioindustry, a wide screening strategy for extra- and intracellular lipases that produce microorganisms has been evaluated. Previous studies conducted by our research group demonstrated that the isolated* A. japonicus* LAB01 was a potential lipase source based on both detection assays of lipase activity in solid and liquid media (data not shown). The present work aims to explore the* A. japonicus* LAB01 lipolytic activity by describing the production, purification, and biochemical characterisation of an extracellular lipase.

## 2. Materials and Methods

### 2.1. Microorganism and Extracellular Lipase Production by* A. japonicus* LAB01 in Shaker Flask Culture

The strain used in this work (*A. japonicus* LAB01) was isolated from urban matured solid compost waste obtained from Coimbra (Brazil, MG) and was kindly provided by the Laboratory of Biochemical Analysis/BIOAGRO/UFV (Brazil). This microorganism was maintained in glycerol and potato dextrose agar (PDA) slants under refrigeration (4°C). Cells were grown on basal medium containing the following (g/L): casein 1.0, NaNO_3_ 1.0, K_2_HPO_4_ 1.52, MgSO_4_ 7H_2_O 0.52, and KCl 0.52, adjusted to pH 6.0, and supplemented with sunflower oil 1.0% (v/v). Cells were grown with shaking at 30°C (200 r.p.m.) for 96 h in 500 ml Erlenmeyer flasks containing 100 ml medium. The inoculum was prepared by transferring eight discs (0.6 cm in diameter) from PDA plate, after growth of the fungus for 96 h at 30°C. To test the effect of immobilised cells on the enzyme secretion, 1 gram of 6 mm cubes reticulated polyurethane foam was added to each flask before autoclaving and the fermentations were incubated as described above. These flasks were incubated at 30°C for 96 h on a reciprocal shaker (200 oscillations/min). When the cells were immobilised, 1 gram of 6 mm cubes reticulated polyurethane foam was added to each flask before autoclaving. The cultivated cells were separated from the culture broth by filtration using Whatman qualitative paper (number 1). The supernatant was considered crude enzyme and was used for the analytical assay. The immobilised cells were washed with tap water and dried at room temperature.

The article "Lipolytic Potential of Aspergillus japonicus LAB01: Production, Partial Purification, and Characterisation of an Extracellular Lipase" was published in 2014. Journal: Biomed Res Int.

### 2.2. Assay of Lipase Activity in Aqueous and Nonaqueous Medium

The lipase activity was measured with a modified spectrophotometric method using p-nitrophenyl palmitate (p-NPP) as a substrate. For the hydrolytic assay, the substrate solution was prepared by mixing 1 mL of solution A (90 mg of p-NPP dissolved in 30 mL 2-propanol) and 9 mL of solution B (90 mM Tris-HCl buffer (pH 8.0); 2.0% Triton X-100; and 0.2% gum arabic). The enzyme-substrate mixture was incubated at 37°C for 5 minutes, and the change in the absorbance was measured at 410 nm in kinetic mode using a microplate reader Varioskan flash and in special cases Shimadzu UV-160A (tests were carried out in temperature higher than 45°C). The molar extinction coefficient of p-nitrophenol (p-NP) was estimated to be 1.27 × 10^3^ M^−1^ *·*cm^−1^. One enzyme unit (U) was defined as the lipase activity that liberated 1 nmol of p-NP per millilitre per minute under the standard assay conditions. For the transesterification assay, methanol and ethanol were used as acyl donors according to Teng and Xu [19].

### 2.3. Lipase Partial Purification

The fermented broth was filtered to obtain a clear supernatant, which was concentrated using ammonium sulphate precipitation at 60% saturation and 4°C with constant stirring overnight. The precipitated protein was collected by centrifugation at 10,000 ×g per 15 minutes and dissolved in a minimum volume of 20 mM Tris-HCl buffer at pH 8.0. The concentrated sample was applied to a Superose 12 HR 10/30 column coupled with the FPLC (fast protein liquid chromatography) system preequilibrated with 20 mM Tris-HCl buffer and pH 7.9 and a flow rate of 30 mL/h. The column was then washed with the same buffer until the flow-through fractions showed no lipase activity. The active fractions were pooled and concentrated by freeze-drying. This concentrated fraction was stored at 20°C until further use. The protein content was estimated using the Bradford reagent as previously described [20, 21].

The article "Lipolytic Potential of Aspergillus japonicus LAB01: Production, Partial Purification, and Characterisation of an Extracellular Lipase" was published in 2014. Journal: Biomed Res Int.

### 2.4. Gel Electrophoresis and Zymography

The lipase molecular mass was determined by SDS-PAGE using a Laemmli system [22] with 12.5% acrylamide. The proteins were stained with a silver stain [23, 24]. For the zymographic analysis, the gel was incubated at 4°C with 100 mL of Tris-HCl buffer (pH 7.9, 20 mM) plus serum albumin (1% w/v) after running to promote protein folding. The gels were incubated for at least 4 hours with solution replacement every 30 minutes. The zymographic analysis was performed based on the lipase hydrolytic and synthetic activity using tributyrin [25], oleic acid, and dodecanol as substrates [26].

### 2.5. Partial Purified Lipase Biochemical Characterisation

All tests to characterise the lipases were conducted in triplicate using the enzyme pool obtained from the purification route described above. Methodologies were designed according to enzymatic characterisation studies employed for lipases from others sources [13, 27–31].

#### 2.5.1. Storage Stability of Crude Enzyme Determination

The storage stability of crude lipase was examined by conserving the cell-free culture supernatant at different temperatures: freezer (−20°C), ultrafreezer (−80°C), fridge (4°C), and room temperatures (22–26°C). The lipase activity was measured every 7 days with a standard pNPP-hydrolysing assay.

#### 2.5.2. pH Effect on Enzyme Activity and Stability

The pH stability was studied by incubating the purified enzyme for 90 min at 30°C in various buffers: 100 mM citrate phosphate buffer (pH 3.0–6.0), 100 mM sodium phosphate buffer (pH 7.0), 100 mM Tris-HCl buffer (pH 8.0-9.0), and 100 mM glycine-NaOH buffer (pH 10.0). The residual hydrolytic activity was then assessed under standard assay conditions using p-NPP as substrate at 37°C and pH 8.0. The optimal pH for the enzyme was determined by measuring the lipase activity using different pH levels for solution B (pH 7–9.5) at 37°C.

#### 2.5.3. Temperature Effect on Enzyme Activity and Stability

The optimal enzyme temperature was determined by assessing the enzymatic kinetics described above at temperatures ranging from 20 to 60°C. The results of this assessment were used to investigate the enzyme thermal stability in that condition by incubating the purified enzyme for 12 h followed by measuring the residual activity.

The article "Lipolytic Potential of Aspergillus japonicus LAB01: Production, Partial Purification, and Characterisation of an Extracellular Lipase" was published in 2014. Journal: Biomed Res Int.

#### 2.5.4. Organic Solvents, Ions, and Detergents Effect on Lipase Stability/Activity

Various effectors, including pure or water-mixed organic solvents (methanol, ethanol, isopropanol, acetone, acetonitrile, toluene, and hexane), ionic solutions prepared in 200 mM Tris-HCl (pH 8.0) buffer (K^+^, Li^+^, Mg^2+^, Ca^2+^, NH_4_^+^, Ni^2+^, Na^+^, Cu^2+^, and Al^3+^), and detergents (1% w/v) (SDS, Tween 80, Triton X-114, and Triton X-100) were added at a proportion of 1 : 1 (v/v) to the purified lipase and incubated in an Eppendorf ThermoMixer (150 rpm) for 90 minutes at 30°C. The lipase activities of the sample without any organic solvent, ions, or detergent were taken as the control (100% of activity). The residual activity was measured with a p-NPP spectrophotometric assay at 37°C and pH 8.0.

#### 2.5.5. Substrate Specificity

The enzyme substrate specificity was investigated by using p-nitrophenyl fatty acid esters of different chain lengths (p-nitrophenyl acetate (C2), p-nitrophenyl butyrate (C4), p-nitrophenyl octane (C8), p-nitrophenyl laurate (C10), p-nitrophenyl myristate (C14), and p-nitrophenyl palmitate (C16) as substrates). The lipase activity was assayed under standard conditions and various preparations of solution A.

#### 2.5.6. Kinetics Parameters Determination

The apparent kinetic parameters (K_M_, *V*_max⁡_, and *K*_cat_) of the partial purified lipase were calculated using a Michaelis-Menten hyperbola direct regression obtained experimentally with the SigmaPlot (v.10) software. The assays were carried out according to the standard reaction using p-nitrophenyl palmitate (C16) as substrate at concentrations varying from 0 to 1.4 mM.

### 2.6. Vegetable Oils Hydrolysis

The hydrolytic activity of crude extracellular lipase from* A. japonicus* LAB01 was determined on emulsified vegetable oils (corn, sunflower, soybean, olive, canola, pequi, almond, macauba, and sesame), according to Soares et al. [32]. The formed fatty acids were titrated with 20 mmol*·*L^−1^ sodium hydroxide solution in the presence of phenolphthalein as indicator. One international unit (IU) of activity was defined as the amount of enzyme that liberates 1 *μ*mol free fatty acid per minute under the assay conditions.

## 3. Results and Discussion

### 3.1. Comparison of Extracellular Lipase Production between Suspension and Immobilised Cells

Supernatants collected after culturing cells in suspension and immobilised into polyurethane foam significantly differed in extracellular lipase activity. For the cell suspension, the lipase activity on supernatant was more than three times greater than the activity obtained for immobilised cells, 28.04 ± 3.11 and 8.09 ± 0.82 (U/mL), respectively. The reduction in lipase secretion during fermentation using immobilised biomass has been attributed to changes in the cell morphology, which can strongly inhibit the secretion of lipase to the medium [33]. Hama et al. [33] showed that the extracellular lipase activity of* Rhizopus oryzae* immobilised cells was approximately half that of suspension cells. Conversely, the intracellular lipase activity of immobilised cells was much higher than that of the suspension cells. Cell immobilisation occurred as a consequence of natural fungi growth, and the liquid media did not contain mycelia mass that had exited the support. The fungi grew into the pores, forming a web biomass that strongly adhered to the support and showed intracellular lipase activity (3.69 ± 0.5 U/g). This result is interesting because it reveals that the lipolytic potential of our strain is not limited to enzyme secretion. The use of intracellular lipases as immobilised biomass has become a promising alternative to catalyse organic reactions, especially for biodiesel production.

The article "Lipolytic Potential of Aspergillus japonicus LAB01: Production, Partial Purification, and Characterisation of an Extracellular Lipase" was published in 2014. Journal: Biomed Res Int.

### 3.2. Extracellular Lipase from* A. japonicus* LAB01 Acting in Organic Medium Performance

To test the catalytic efficiency of extracellular lipase from* A. japonicus* LAB01 to act in an organic medium, the supernatant was concentrated and completely dried, which prevented a parallel hydrolysis reaction. The enzyme could catalyse the pNPP transesterification using anhydrous methanol and ethanol as the acyl donor group, with 23.60 ± 0.93 and 30.336 ± 2.60 (U/mL) of enzymatic activity, respectively. The enzyme more efficiently catalysed the hydrolysis reaction with an activity of 199.5 ± 10 (U/mL). In general, the catalytic activity displayed by enzymes in neat organic solvents is far lower than in water [19, 20, 30, 34]. This difference has been attributed to the enzyme's decreased flexibility, denaturation by contact with the organic solvent, and diffusion effects [30]. This difference could also be due to the drying step effect. For example, lyophilisation can significantly change the enzyme structure to reduce the enzymatic activity in organic solvents [34]. The obtained data agree with those observed for lipases from* Pseudomonas aurantiogriseum*. This enzyme exhibited an activity of 312.3 (U/mg) and 13.6 (U/mg) on the pNPP substrate in organic and aqueous media, respectively [30]. Commercial lipases from* Candida rugosa*,* Penicillium* sp., and pig pancreas demonstrated the absence of p-NPP transesterification in the presence of ethanol [19]. However, the enzymes effectively catalysed the substrate hydrolysis. In fact, the hydrolytic and synthetic activities of lipases do not directly correlate. These preliminary results demonstrated the versatility of reactions with lipase from* A. japonicus* LAB01 and suggest that this enzyme could be applied in the transesterification catalysis of natural substrate (oil and fat) to produce biodiesel.

The article "Lipolytic Potential of Aspergillus japonicus LAB01: Production, Partial Purification, and Characterisation of an Extracellular Lipase" was published in 2014. Journal: Biomed Res Int.

### 3.3. Lipase Partial Purification

*A. japonicus* LAB01 lipases were purified using (NH_4_)_2_SO_4_ selective precipitation (60%) followed by gel filtration chromatography (Table 1). After two steps of purification, the lipase exhibited 3.5 × 10^4^ U*·*mg^−1^ specific activity and 2.91-fold purification with an overall yield of 44.2%. The protein purification step profile showed a strong protein band with a molecular mass between 25 and 35 kDa estimated by SDS-PAGE (Figure 1). The zymographic analysis using tributyrin, oleic acid, and dodecanol as substrates revealed hydrolytic and synthetic activities based on bands that coincided with the migration of the principle protein (Figure 2). The partially purified lipase molecular mass was estimated to be approximately 25 kDa on SDS-PAGE. Most of the known* Aspergillus* sp. lipases reportedly have molecular masses in the range of 29−70 kDa [7, 10]. Another lipase from* A. japonicus* was purified by combining anion exchange (Q-Sepharose) and gel filtration (Sephadex G-100) chromatography by 3.44-fold with a 4.53% yield and a specific activity of 480 U/mg protein. The molecular weight of the enzyme was 43kDa according to SDS-PAGE [35]. Other lipase isoforms also differ in their molecular mass, such as those observed on* Aspergillus niger*. Two lipases from* A. niger* MZKI A116 were isolated by acetone precipitation followed by ion-exchange chromatography. The molecular weights were 43 kDa and 65 kDa, with isoelectric points of pH 4.1 and 4.2, respectively [36]. Recently, a novel lipase produced by the same fungus was found [37]. An extracellular lipase from the* Aspergillus niger* NCIM 1207 strain was purified by homogeneity using ammonium sulphate precipitation followed by phenyl-sepharose and Sephacryl-100 gel chromatography to yield a monomeric protein of 32.2 kDa.

### 3.4. Biochemical Characterisation of Lipases from* A. japonicus* LAB01

#### 3.4.1. Crude Lipase Storage Stability Determination

To verify the storage stability of the crude extract that contained extracellular lipase from* A. japonicus* LAB01, the supernatant was stored under the following conditions: refrigerator (4°C), room temperature, freezer (−20°C), and ultrafreezer (−80°C), and the enzyme activity was measured weekly for 1 month. As shown in Figure 3, the enzyme retained at least 40% of its initial activity under the tested temperature conditions. The best supernatant storage condition was found to be in the ultrafreezer (−80°C). The enzyme retains approximately 80% of its initial activity (%) after 4 weeks of storage. Good storage stability for lipase from* A. japonicus* LAB01 is a prerequisite for laboratory bench scale tests and for its future industrial application. Similar results were found for an extracellular* Lactobacillus plantarum* lipase, which was stable at −80°C for 4 weeks, retaining 90% of its initial activity [38].

The article "Lipolytic Potential of Aspergillus japonicus LAB01: Production, Partial Purification, and Characterisation of an Extracellular Lipase" was published in 2014. Journal: Biomed Res Int.

#### 3.4.2. Effect of pH on Lipase Stability and Activity

The lipase stability was evaluated in the pH range of 3.0 to 10.0 using different buffers at the same concentration (100 mM) (Figure 4). The enzyme remained stable from pH 5.0 to 9.0 during preincubation for 90 min at 30°C, where the enzyme retained at least 80% of its initial activity. Furthermore, increasing or decreasing the pH values dramatically reduced the enzyme stability. The* A. japonicus* LAB01 lipase was more active at slightly alkaline pH values, and the optimal pH was 8.5, which is similar to the values reported for lipases from* A. carneus* [13]. The purified enzyme from our strain did not show differences in the optimum pH and pH stability; consequently, the lipase could be considered a resistant alkaline lipase. Alkaline lipases are required for applications in the detergent industries, suggesting a possible use in this area. The majority of the lipases of* Aspergillus* origin showed maximum activities in neutral or near neutral pH values (6.0–7.5), such as those obtained from* A. japonicus* [35],* A. niger* MTCC 2594 [39],* A. nidulans* [40],* A. niger* F044 [41],* A. awamori* [42],* A. niger* MYA135 [27], and* A. terreus* [43].* A. niger* NCIM 1207 lipase, which exhibited an optimum acidic pH of 2.5, was an exception to this rule [37].

#### 3.4.3. Temperature Effect on Lipase Activity and Stability

The purified lipase was active in the temperature range of 20–45°C, with maximal activity at 45°C. Its activity sharply decreased above the optimum temperature (Figure 5). The characteristics of* A. japonicus* LAB01 lipase were not consistent with those of others found in* Aspergillus* genus, including* A. niger* MTCC 2594 [39],* A. carneus* [13], and* A. niger* MYA135 [44]. In all of these cases, the optimum temperature was 37°C, and the enzymes were not very active at temperatures above 40°C. The recombinant* A. fumigatus* lipase, whose optimal temperature was 65°C, constitutes an exception. However, this enzyme was not stable at this temperature, losing almost 100% of its activity after 1 h of incubation [29]. The thermal stability profile of* A. japonicus* LAB01 lipase indicated that this enzyme was stable at 45°C for at least 3 h, retaining 70% of its original activity. The high thermal stability of the enzyme is similar to that found for the thermostable lipases obtained from* R. homothallicus*, which had a half-life equal to 0.72 hours at 50°C [45]. The thermal stability of lipase from our strain indicates its potential application in the modification of vegetable oils, mainly oils that have high melting points, which are solid at room temperature. In general, fungal lipases are not stable at temperatures above 40°C. Some studies have reported lipases with moderate thermostability, as observed for* P. wortmanii* lipase, which retained 90 and 55% of its initial enzymatic activity after 60 min of incubation at 45 and 50°C, respectively [46].* P. cyclopium* lipase was stable for 1 hour when incubated at 30°C and only lost 10% of its activity after 1 hour of incubation at 35°C [47].* P. crustosum* lipase lost 75% of its enzymatic activity after incubation for 1 hour at 45°C [48].

The article "Lipolytic Potential of Aspergillus japonicus LAB01: Production, Partial Purification, and Characterisation of an Extracellular Lipase" was published in 2014. Journal: Biomed Res Int.

#### 3.4.4. Substrate Specificity

The specificity of lipases is related to the carboxylic acid ester type and sets them apart from conventional chemical catalysts, especially for their application in structured triacylglycerol synthesis, chemical reaction intermediates, and resolution of chiral compounds. Therefore, this property is of great industrial importance and depends on the enzyme source. The specificity of the partially purified* A. japonicus* LAB01 lipase for chain length was evaluated based on the initial hydrolysis rate, employing acyl esters of p-nitrophenyl (pNP) with carbon chain sizes ranging from C2 to C16: acetate (C2, pNPA), butyrate (C4, pNPB), caprylate (C8, pNPC), decanoate (C10, pNPD), laurate (C12, pNPL), myristate (C14, pNPM), and palmitate (C16, pNPP). The specific profile showed that the enzyme activity positively correlated with the length of the substrate carbon chain (Table 2). The enzyme showed little activity on short-chained acyl esters, such as pNPA (C2) and pNPB (C4), and had the highest activity on pNPM (C14) (Table 2). The preference for pNPM (C14) substrate was also observed for lipase from* Serratia marcescens* ECU1010 [49]. Conversely, another lipase purified from* A. japonicus* exhibited a preference for the pNPP (C16) substrate, and less than 80% residual activity was found on pNPM [35]. Most of the described microbial lipases are more active in the cleavage of long or medium chain fatty acid substrates, as noted for lipases mentioned before as well as lipases from* A. carneus, Staphylococcus aureus,* and* Penicillium aurantiogriseum*, which showed a preference for pNPD substrate (C10) [13, 30, 50];* A. niger* MYA lipase prefers pNPO (p-nitro substrate) (C18) [27];* P. crustosum* lipase prefers pNPL (C12) [48]. However, a new type of lipase gene, which was cloned from the genomic DNA of* A. fumigatus* (CGMCC 2873), showed extremely high hydrolytic activity toward p-short-chain nitrophenyl esters, such as pNPA (C2) [29].

The article "Lipolytic Potential of Aspergillus japonicus LAB01: Production, Partial Purification, and Characterisation of an Extracellular Lipase" was published in 2014. Journal: Biomed Res Int.

#### 3.4.5. Ions Effect on Lipase Stability

Lipases are known not to require cofactors to act; however, metal ions significantly affect the stability of lipases. Some metal ions interact with the enzyme surface charge, affecting the ionization of some amino acid residues, changing the enzyme conformation, and rendering it less stable and/or altering its activity. This process is known as ion toxicity [51]. The behaviour of* A. japonicus* LAB01 lipase in the presence of some ions was investigated using chloride or sulphate salts of each ion at a concentration of 10 mM in Tris-HCl buffer (pH 8, 200 mM) at 30°C for 90 minutes. The results showed that K^+^, Na^+^, Ca^2+^, Mg^2+^, NH_4_^+^, and Li^+^ ions slightly increase the lipase activity up to 12% or exerted no effect on the activity, whereas lipase activity was inhibited by Cu^2+^, Ni^2+^, and Al^3+^ (Table 3). Enzymes, such as lipases, need to be stable at high salt concentrations in some cases, such as when a lipase is used in a waste processes, like the continuous removals thin layers of fats and oils from the surface of aerated tanks to permit oxygen transportation. Wastewater sources and their ion contents constitute another variable in this process. Furthermore, ion-exchange chromatography is a common step in purification methods used in lipase purification strategies, and adding specific ions to the buffer can increase the yield. Metal ions also affect lipase substrates; Hasan et al. [9] reported that these metals would form complexes with ionised fatty acids, changing their solubility and behaviour at the interfaces. The stability of the lipase depends on its source and even the isoforms. The addition of 2 mM metal ions in a 50 mM Tris-HCl buffer (pH 8.0) at 30°C for 0.5 h did not increase the activity of lipase from* A. fumigatus*. The enzyme was stable (residual activity > 95%) in Ca^2+^ and Ni^2+^. Conversely, Cu^2+^ and Zn^2+^ inhibited the lipase (residual activity < 50%) [29]. Incubation with 10 mM Ba^2+^ at 30°C for 30 minutes stimulated the activity of* A. terreus* var. africanus lipase by 52%, while Cu^2+^, Fe^2+^, Fe^3+^, Hg^2+^, and K^+^ completely inhibited the enzyme [43].

#### 3.4.6. Detergents Effect on Lipase Stability

Detergents have been used in some lipase activity assay protocols for immobilisation and biotransformation and may have both a positive and a negative effect on the enzyme activity, which depends on the concentration or detergent nature. As shown in Table 4, ionic surfactants, such as Tween 80 and Triton X-100 at 1% (v/v) decreased the lipase activity by 70 and 12%, respectively. Similar to lipases from* A. fumigatus*, which were unstable in SDS (0.1% v/v) [29], the* A. japonicus* LAB01 lipase was sensitive to the anionic surfactant SDS, which completely inhibited the lipase hydrolytic activity. The negative effects of detergents on the stability of* A. japonicus* LAB01 lipase can be attributed to the competition between the substrate and detergent for the adsorption site in the enzyme or distortion in the enzyme structure [52, 53]. The concentration of the detergent evaluated may also exert negative effects. Studying the stability of free and immobilised lipases from* Pseudomonas fluorescens* [53] showed that the activity/detergent concentration curve reached a maximum activity value and began to decrease as the detergent concentration increased, in many instances even below the initial value.

The article "Lipolytic Potential of Aspergillus japonicus LAB01: Production, Partial Purification, and Characterisation of an Extracellular Lipase" was published in 2014. Journal: Biomed Res Int.

Conversely, the lipase from* Spirulina platensis* was active in the presence of 0.1% Triton X-100 or 0.5 mM SDS, showing residual activities (%) of 121 and 103, respectively [54]. The large increase in the lipase activity, which was mainly observed for the immobilised form, can be attributed to the potential of these surfactants to break the lipase-lipase dimmers and alter the closed-open equilibrium of the individual lipase molecules [53, 55]. Moreover, the presence of detergents also improved the enantioselectivity of lipases. For example, the enantioselectivity of* Pseudomonas fluorescens* immobilised in glyoxyl agarose increased from 40 to more than 100 in the (±)-2-hydroxy-4-phenylbutyric acid ethyl ester hydrolysis when using 0.1% (v/v) hexadecyltrimethylammonium bromide (CTAB) [53].

#### 3.4.7. Solvent Effect on Lipase Stability

Reaction media that consist of organic solvents can greatly expand the lipase-catalysed transformation repertoire, where numerous reactions might be used by synthetic and polymer chemists with high selectivity [34]. Furthermore, solvents affect the catalytic proprieties, such as the selectivity lipases, and increase the substrate solubility, eliminating mass-transfer barriers for substrates [56]. Hence, the stability and activity of lipases in solvents are considered an important investigation point. To study effects of organic solvent on* A. japonicus* LAB01 lipase, the enzyme was incubated with different solvents at 30°C for 90 min, and the residual enzymatic activity was determined at assay conditions. As shown in Table 5, the enzyme was activated in pure nonpolar solvents, showing 100% and 137% residual activity in toluene and hexane, respectively. Toluene has a strong antimicrobial potential; thus, it constitutes an alternative method to preserve* A. japonicus* LAB01 lipases during storage. The enhancement of enzyme activity due to solvents could be attributed to lipase disaggregation, some structural changes in the enzymes (maintaining the lipase on its open conformation), and even modification at the oil-water interface to facilitate enzymatic action [57].

The article "Lipolytic Potential of Aspergillus japonicus LAB01: Production, Partial Purification, and Characterisation of an Extracellular Lipase" was published in 2014. Journal: Biomed Res Int.

Conversely, the lipase molecule was unstable in pure polar solvents, completely losing its activity in acetone and acetonitrile. Regarding the solvents employed in biodiesel production, the enzyme was more stable in a methanol solution, mainly at 50% (v/v) concentration, than in ethanol and propanol. The effect of the solvent polarity does not explain this finding; rather, this effect is likely due to the similar sizes of the water and methanol molecules, which can decrease the distortion in the three-dimensional structure of the protein. The enzyme was sensitive to the increased alcohol concentration, almost losing activity at increasing alcohol concentrations up to 75% (v/v).

In general, hydrophobic solvents are usually superior to hydrophilic ones as enzymatic reaction media because the latter are likely to tightly strip the bound water (which is essential to the catalytic properties and structure) from the enzyme molecules [34]. In fact, lipases are diverse in their sensitivity to organic solvents, but polar solvents are generally agreed to be more destabilising than nonpolar solvents, as has been demonstrated for lipases from* Staphylococcus* sp. [58],* Penicillium* sp. DS-39 (DSM 23773) [59], and* Idiomarina* sp. W33 [60].

Yang et al. [56] studied the effect of organic solvents on the conformation of recombinant* Candida antarctica* lipase (CALA). Treating CALA with acetonitrile increased the *α*-helical content and decreased the random coil content. The changes in the secondary structure of the enzyme were mainly responsible for the variance of the catalytic activity, which allowed this enzyme to be used for organic synthesis and chiral resolution. However, no obvious relationships could be established for any distinctive change in activity caused by the types of solvents.

#### 3.4.8. Kinetics Parameters Determination

The apparent kinetic parameters for partially purified lipase were obtained from a rectangular hyperbola equation using the SigmaPlot software (version 10.0) (Figure 6). It yielded apparent K_M_ and *V*_max⁡_ values of 0.13 mM and 12.58 *μ*M*·*min^−1^, respectively, for p-NPP as a substrate. Similar kinetic parameters were also found for* A. awamori* (0.13 mM) [61] and* A. nidulans* (0.28 mM) lipases [62].

The article "Lipolytic Potential of Aspergillus japonicus LAB01: Production, Partial Purification, and Characterisation of an Extracellular Lipase" was published in 2014. Journal: Biomed Res Int.

### 3.5. The Application of Lipases to Catalyse Vegetable Oil Hydrolysis

Lipases from* A. japonicus* LAB01 could hydrolyse all commercial oils tested and activities were expressed as percent of activity against canola oil. The enzyme preferentially catalysed canola and almond oils, showing yields of 100 ± 0.84 and 83 ± 0.73%, respectively. For other oils evaluated, the yields (%) were: corn oil (62 ± 0.01), pequi oil (55 ± 0.42), sesame oil (52 ± 0.02), sunflower oil (52 ± 0.01), soybean oil (48 ± 0.42), and olive oil (38 ± 0.42). As mentioned above, the specificity of lipases depends on their source. Rice bran oil and sardine oil were effectively hydrolysed by* Cryptococcus* sp. S-2 lipases with 80.2 and 76% activity on triolein [63].* Rhizopus oryzae* lipases more efficiently hydrolysed olive oil, with a yield of 48% against trioctanoin [31]. From a biotechnological point of view, the use of lipases in the oleochemical industry is adequate because is an energy-saving process and unsaturated fatty acids can be produced without oxidation [64].

## 4. Conclusion

The lipolytic potential of* A. japonicus* LAB01 was demonstrated based on its ability to produce extracellular and intracellular lipases. The extracellular lipase from* A. japonicus *LAB01 showed versatile and interesting catalytic properties: it may act in aqueous and nonaqueous media, exhibiting maximum activities at alkaline pH values and increased temperatures (45°C), and it is compatible with processes used to modify fats and oils. Furthermore, the enzyme showed good stability when placed in contact with organic solvents, salt, and detergents. Future developments in the optimisation of extra- and intracellular lipase production and biotechnological applications for this lipase will be interesting to follow.

## Figures and Tables

**Figure 1:** SDS-PAGE of purified lipase from* A. japonicus* LAB01. Lane 1: molecular mass markers; Lane 2: purified lipase after (NH_4_)_2_SO_4_ precipitation; Lane 3: purified lipase after gel filtration.

**Figure 2:** Zymographic analysis after SDS-PAGE gel electrophoresis of lipase from* A. japonicus* LAB01. Lane 1: lipase activity towards tributyrin; Lane 2: lipase activity towards oleic acid and dodecanol; Lane 3: molecular mass markers.

**Figure 3:** Storage stability of crude lipases from* A. japonicus* LAB01. Freezer (−20°C) (diamond), ultrafreezer (−80°C) (triangle), fridge (4°C) (circle), and room temperature (square).

The article "Lipolytic Potential of Aspergillus japonicus LAB01: Production, Partial Purification, and Characterisation of an Extracellular Lipase" was published in 2014. Journal: Biomed Res Int.

**Figure 4:** Effects of pH on the stability (a) and activity (b) of* A. japonicus* LAB01 lipase. (a) Partially purified lipase samples were incubated for 90 min at 30°C in the presence of different buffers (100 mM): citrate phosphate (pH 3.0–6.0), sodium phosphate (pH 7.0), Tris-HCl (pH 8.0-9.0), and glycine-NaOH (pH 10.0), and the residual activity was measured using pNPP at pH 8.0 and 37°C. (b) Partially purified lipase samples were assayed in buffers B from pH 7.0 to 9.5 using pNPP as substrate at 37°C.

**Figure 5:** Effects of temperature on stability (a) and activity (b) of the partially purified* A. japonicus* LAB01 lipase. (a) Temperature stability profile was determined by measuring the residual activity at pH 8.0 and 37°C after incubating the lipase at 45°C for 720 min. (b) Optimal temperature was determined by measuring the enzyme activity at different temperatures at pH 8.0.

**Figure 6:** Michaelis-Menten hyperbola plot for K_M_ and *V*_max⁡_ values of* A. japonicus* LAB01 lipase in the presence of various concentrations of p-NPP.

**Table 1:** Summary of purification of extracellular lipase from *A.  japonicus* LAB01.

Purification step	Volume (mL)	Total protein (mg)	Specific activity (U*·*mg^−1^)	Total activity (U*·*L^−1^)	Fold purification	Yield (%)
Supernatant	410	13.12	9.20 × 10^3^	1.21 × 10^5^	1.00	100
Ammonium sulphate precipitation (60%)	15	4.76	2.69 × 10^4^	1.28 × 10^5^	2.92	106
Gel filtration chromatography (Superose 12 HR)	11	1.49	3.59 × 10^4^	5.33 × 10^4^	3.91	44.2

**Table 2:** Substrate specificity of *A. japonicus* LAB01 lipase for various acyl esters of p-nitrophenyl (pNP).

Substrate	Residual activity (%)
C2 (pNPA)	14.18 ± 1.61
C4 (pNPB)	23.42 ± 1.20
C8 (pNPC)	45.21 ± 1.59
C10 (pNPD)	48.10 ± 3.73
C12 (pNPL)	70.42 ± 6.37
C14 (pNPM)	107.09 ± 0.41
C16 (pNPP)	100 ± 0.43

Activities are expressed as per cent of activity against pNPP. The assays were carried out in pH 8.0 at 37°C, preparing different formulations of solution A as described above. Assays were performed in triplicate and mean values are reported.

**Table 3:** Effect of ions on the activity/stability of the lipase from *A.  japonicus* LAB01.

Ions	Residual activity (%)
Mg^2+^	112.97 ± 3.73
Li^+^	109.22 ± 0.91
NH_4_^+^	104.03 ± 2.98
Na^+^	107.61 ± 2.27
Ni^2+^	70.42 ± 1.72
Cu^2+^	59.84 ± 1.27
K^+^	103.22 ± 2.36
Ca^2+^	98.03 ± 1.58
Al^3+^	42.11 ± 5.08

Lipase samples were incubated in each ionic solution prepared in 200 mM Tris-HCl (pH 8.0) buffer at 30°C for 90 min. The remaining lipase activity relative to the non-ion containing control was determined on pNPP substrate at pH 8.0 and 37°C. Values are the average of assays carried out in triplicate.

**Table 4:** Effect of detergents on the activity/stability of the lipase from *A. japonicus* LAB01.

Detergent	Residual activity (%)
Triton X-100	88.80 ± 1.16
Triton X-114	34.05 ± 2.65
Tween 80	32.50 ± 1.34
SDS	0

Lipase samples were incubated with each detergent (1% v/v) at 30°C for 90 min. The remaining lipase activity relative to the non-ion containing control was determined on pNPP substrate at pH 8.0 and 37°C. Values are the average of assays carried out in triplicate.

The article "Lipolytic Potential of Aspergillus japonicus LAB01: Production, Partial Purification, and Characterisation of an Extracellular Lipase" was published in 2014. Journal: Biomed Res Int.

**Table 5:** Effect of organic solvents on the activity/stability of the lipase from *A. japonicus* LAB01.

Solvents	Residual activity (%)
Hexane	137.1 ± 4.71
Toluene	100.9 ± 4.70
Acetonitrile	0
Acetone	0
Methanol (25% v/v)	98.48 ± 0.97
Methanol (50% v/v)	108.09 ± 0.34
Methanol (75% v/v)	13.10 ± 0.87
Ethanol (25% v/v)	90.71 ± 3.89
Ethanol (50% v/v)	12.65 ± 1.65
Ethanol (75% v/v)	4.03 ± 0.03
Isopropanol (25% v/v)	70.65 ± 0.25
Isopropanol (50% v/v)	2.05 ± 0.19
Isopropanol (75% v/v)	1.64 ± 0.06

Lipase samples were incubated with organic solvents at 30°C for 90 min. The remaining lipase activity relative to the non-solvent containing control was determined on pNPP substrate at pH 8.0 and 37°C. Values are the average of assays carried out in triplicate.
